RETRACTED

# The bibliometric analysis of previous twenty- five years’ literature: A microfinance review

**DOI:** 10.1016/j.heliyon.2024.e24979

**Published:** 2024-01-19

**Authors:** Kashif Beg, B. Padmapriya, Syed Noorul Shajar, Md. Moneef Ahmad, Abdul Ghani Faiyyaz

**Affiliations:** a School of Business (VSB), VIT-AP University, Andhra Pradesh, India; b Department of Commerce, NMIMS, Hyderabad, India; c Department of Commerce, School of Social Sciences and Languages, VIT, Vellore, India; d Sharda School of Business Studies, Sharda University, Greater Noida, Uttar Pradesh, India; e Department of Commerce, SRM Sikkim University, Sikkim, India

**Keywords:** Bibliometric analysis, Citation analysis, Literature review, Microfinance, Most cited documents, Three field plot, Trend topic, Word cloud

## Abstract

The tremendous increase in publications in Microfinance since 2000 has highlighted need for and importance of innovative techniques to present big data in this field in a most informative, scientific, and summarized manner. The study highlights the trends and patterns of Microfinance literature by revealing what has been done and what could be done in future. The study comprises of 1429 microfinance publications extracted from the Scopus database. The authors adopt bibliometric analysis through open software application R and network analysis techniques using Gephi AND VOS viewer software. The study adds a valuable contribution to the field of Microfinance by distinctively summarizing the important literature. It identifies global academic research trends and provides insights about trending topics, highly cited literature, authors, countries, collaboration network, word cloud, citation analysis, etc. Finally based on extensive literature survey through bibliometric analysis. The study highlights about the scope of future research in Microfinance.

## 1 Introduction

Microfinance has proven to be crucial to a nation's holistic growth and development. Providing financial services to the deprived and low-income members of society promotes extensive financial services penetration in an economy and consequently aids in growth [1]. In the 1990s, microfinance—the provision of financial services to the underprivileged and the needy segment of society with a small number of deposits and loans became well known. The Grameen Bank model developed by Mohammad Yunus, who received the Nobel Peace Prize in 2006 for it, led to the reduction of poverty and the empowerment of low-income women. The Grameen Bank approved over 6.5 million dollars in loans over the past 20 years, constantly keeping its loan repayment percentage above 98 %. The loans were approved without collateral [2]. The application of microfinance and its potential to combat social and financial inequalities are growing research areas [3].

RETRACTED

Microfinance is a problem for Muslim countries and their citizens. The lack of ethical and moral values in microfinance through riba (interest) based financing is a major concern [4]. Rokhman [5] found that Islamic microfinance emerged as an alternative. This facility can cover the purpose of microfinance based on Islamic values. As Riba is ban as per Islamic law.

Islamic microfinance has grown significantly alongside mainstream microfinance. Islamic microfinance seeks to enhance the well-being of the poor by increasing earnings and consumer spending and improving living standards through Shariah principles [6]. The study applied a bibliometric tool to determine the research gaps, trends, and gives a direction for future research. The study uses a methodical scientific approach to gather the data required for the researchers and to identify their future research plan. Without any prejudice, the bibliometric and citation analysis highlights to find significant studies and researchers. A detailed overview of the most important studies is provided to summarize the findings, which might be helpful to academicians interested in microfinance research.

An abundance of literature has been published in the field of Microfinance in the last three decades. The traditional review studies in the area of Microfinance are making it difficult for researchers to trace the relevant and important contributions [7]. This literature survey summarizes the literature on microfinance through bibliometric analysis and network analysis. Bibliometric analysis is the new technique to analyze the bibliographic data of published literature to describe patterns of publication within a given field. The objective of this research is to present a structured review of Microfinance literature. The study adds a valuable contribution to the field of Microfinance by providing a summarized picture of important literature from different perspectives which is extremely beneficial for researchers interested in the area of Microfinance. A structured and well-designed review is completely different from the descriptive literature review traditionally investigated by authors [8].

The current work can be divided roughly into five categories. An introduction overview is given in Section 1. Section 2 discusses the relevant literature and review studies of Microfinance. Data and research methods used are highlighted in Section 3. Section 4 demonstrates the data analysis using network analysis and bibliometric analytics tools from various perspectives. Section 5 concludes with recommendations for further research.

RETRACTED

## 2 Literature review

Microfinance not only includes microcredit but also includes small savings, insurance services for the poor, and money transfers. It is recognized as a tool for reducing poverty by assisting micro-entrepreneurs in growing their businesses and boosting their income and assets. Microfinance helps in enhancing the lives of millions of poor people to overcome poverty by augmenting non-financial outcomes like, education, health, food security, women empowerment, and housing as well as financial outcomes like income, saving, and the accumulation of assets like furniture or a sewing machine [9,10,11,12,13,14,15,16,17,18].

Although several research papers cast doubt on the benefits of microfinance. Some studies show more mixed effects, such as improved economic well-being for the poor but not of the poorest [19,3,20,21]. Hulme and Mosley [22] found microfinance had no significant impact in terms of raising income or empowering women. Some studies revealed negative effects like obstacles to sustainable local economic and social development, exploitation of women, suicides, child labor, coercive loan recovery practices etc [23,24,25]. Previous studies revealed that microfinance alone is not much effective as an anti-poverty tool but that it can be used in conjunction with other anti-poverty measures [26,27,28,29,30].

Islamic microfinance is also on the rise in disadvantaged Muslim countries. In terms of efficiency, there was no significant difference between traditional and Islamic microfinance. It is regarded as a successful tool representing his two companies in Islamic finance and microfinance [31]. After finding that Bangladesh's traditional microfinance programs were not successful in reducing poverty due to factors such as religious restrictions and interest-driven borrowing costs, Ashraf [32] argued that Islamic microfinance could help poor Islamic countries. He suggested that it could be an alternative for believers. After extensive review of previous empirical studies and related literature, Abdul-Majeed Alaro and Alalubosa [33] proposed Islamic microfinance as a financial strategy to reduce poverty in Nigeria. In fact, various studies show that Islamic microfinance has a positive impact, especially on improving livelihoods and reducing poverty. For example, Baitul Mar Wat Tamwir (BMT) is an Indonesian Islamic Microfinance Institution (IMFI), which has been shown in several studies to be effective in reducing poverty in this developing country [34,5]. According to Quraisy, Hamzah, and Razzaq [35], 145 borrowers improved their physical and social well-being after participating in BMC [[36], [37], [38], [39], [40]]. all reached similar conclusions.

RETRACTED

### 2.1 Specific review: review studies of microfinance

There are few renowned reviews studies examining the impacts of microfinance [[15], [41], [42], [43], [44], [45], [46]]. Brau and Woller [41] reviewed over 350 articles related to issues of Microfinance institution's sustainability, product and services management practices, clientele targeting, regulation and policy, and impact assessment. The study concluded that the model, and framework in the existing literature might resolve the problem of poverty to a great extent. Sebstad and Chen [46] summarize the key findings from 32 studies regarding the impact of microcredit services on household economic security, individual control over resources, and enterprise stability and growth. The study showed a positive impact of microfinance on educational attainment, school attendance, and school enrolment levels and found some improvement in health and nutrition levels. The study revealed that Microfinance programs effectively reached many poor households but have differential effects on participants and most notably in terms of increase in household and enterprise income and assets. Gaile and Foster [43] reviewed eleven studies carried out in Asia, Africa, and Latin America to identify the impact of microenterprise credit programs. They found that few of the quantitative studies did not adequately focus on selection bias, temporal execution issues, analytical techniques, control methods and sample design. Goldberg [44] comprehensively examined 100 studies released since 1986 to measure the impact of Microfinance. The study disclosed a wide range of evidence that microfinance is a useful tool for increasing income and poverty reduction. A wide range of Microfinance services by MFIs can also improve children's nutrition and school enrolment rates. Odell [15] highlights that impact of microfinance on poverty alleviation and increase in income is ambiguous. The empirical findings regarding impact vary greatly with a short-term increase in investment and expansion of business but not leading to immediate well-being effects. The study investigated the most recent contributions and suggested that Microfinance increases business ownership, investment, and profit. Additionally, the most promising financial instrument was found to be micro saving.

## 3 DATA and research methods

The term Bibliometric review was first introduced by Alan Dritchard in 1969 to denote a new discipline where quantitative methods were employed for measuring and analyzing publication patterns by mathematical and statistical techniques. Van [47] highlights the significance of bibliometric techniques in social sciences. The study focuses on citation flows, the origin of publication, and social sciences reference coverage in terms of citations. To develop well-founded insight and understanding of the various fields of social sciences, the research stresses the underlying dynamics of the social sciences, both in terms of publication and citation culture. In the field of dividend policy, Pinto et al. [48] employed bibliographic analysis. Ali and Bashir [49] has applied bibliometric analysis to asset pricing studies. Firdaus et al. [50] analyzed 1000 articles from the Scopus database by using bibliographic analysis to study the in-depth research pattern of Blockchain. Syed and Bawazir [51] analyzed 3024 financial risk publications of ten years indexed in the web of science by Bibliometric analysis. The study used bibliometric and network analytic tools to emphasize a comprehensive view of microfinance research to identify the gap in the field. The research presents a thorough analysis of the literature in the Scopus database, based on which the most recent research trends are identified and future research potentialities, or uncharted areas, are forecasted. The study followed the procedures outlined in the following subsections.

RETRACTED

### 3.1 Recognition of the perfect search words

Keeping in mind the objective of this study, i.e., to identify the general trends in the field, the research considered almost three decades (1996–2019) to have a clearer view of the trend in microfinance. The Scopus database was searched by using “Microfinance” as the specific keyword. The elementary result generated a list of 2061 research article results. Following Tsay and Shu [52], we specified the command search to "Journals" publications only under "articles and review papers." Further, we limit the documents to the "English" language. In a further refinement, we exclude articles with no author, and thus left with the final 1429 documents. The findings, which included the author's name, abstract, article title, keywords, references, etc., were saved in CSV format. The results were used as the primary source of data for performing systematic literature review.

## 4 Analysis of DATA

Network analysis tools are employed to analyze the latest issues in the Microfinance area to determine the trends and areas. Keywords, journals, and statistics are analyzed through Bibliometric analysis.

### 4.1 Descriptive analyses of ARTICLES

Table 1 highlights the full information about the published papers taken from Scopus. We started by searching the keywords “Microfinance” in article searches in Scopus database. Secondly, we choose research articles from search results so that search items are restricted to only on research papers from search items for the period 1996–2019. In a total of 1429 articles are considered from the period of 1996–2019, out of that 1394 are research articles and 35 review papers. The result shows that 1109 unique keywords and 2314 author keywords are used. The review period lasted 25 years starting from 1996 to 2019 showing average citations of 13.26 per document. The result shows 2197 authors of these articles and 1429 documents 386 are single-authored and 1811 are written by multi authored. Collaboration index indicates that Documents are developed in an average of 2 collaborations institutions.

RETRACTED

**Table 1:** Descriptive analyses of ARTICLES.

Description	Results
Documents	1429
Sources (Journals, Books, etc.)	530
Keywords Plus (ID)	1109
Author's Keywords (DE)	2314
Period	1996–2019
Average citations per document	13.26
Authors	2197
Author Appearances	3046
Authors of single-authored documents	386
Authors of multi-authored documents	1811
Documents per Author	0.65
Authors per Document	1.54
Co-Authors per Documents	2.13
Collaboration Index	1.92

### 4.2 Annual publication growth analysis

Fig. 1 shows a line graph showing the total number of publications in the field of microfinance from 1996 to 2019. It has an increasing rate of 4.2% every year. The years 2017 and 2019 saw the most articles published ever with 157 and 153 articles, respectively. From 18 papers published in 2000 to 153 articles published in 2019, the number of articles published has shown significant increased. The line chart's rising trend suggests that scholars are becoming more interested in investigating this crucial field of study for stakeholders, policymakers, and microfinance regulatory organizations.

**Fig. 1:** Number of articles published each year..

### 4.3 Highly cited ARTICLES

The list of documents and the number of citations are displayed in Table 2. According to the table, the article by Battilana and Dorado [53] that was published in the Academy of Management Journal has received the highest citations. “Building Sustainable Hybrid Organizations: The Case of Commercial Microfinance Organizations” is the title of this document. Others highly cited publications are those by Khandker [54] in the Journal of Economic Literature. Morduch [3] research was published in the World Bank Economic Review. Table 2 displays the total number of publications by both individual and collaborative authors. The list is displayed in the table in decreasing order.

**Table 2:** Highly cited ARTICLES.

Document	Author	Total citations	Year	Journal
Building sustainable hybrid organizations: The case of commercial microfinance organizations.	Battilana J & Dorado S	854	2010	*Academy of M Journal*
The microfinance promise.	Morduch J	839	1999	*Journal of Economic Literature*
Microfinance and poverty: Evidence using panel data from Bangladesh.	Khandker SR	373	2005	*The World Bank Economic Review*
The microfinance schism.	Morduch J	357	2000	*World Development*
Outreach and efficiency of microfinance institutions.	Hermes N	229	2011	*World Development*
Social capital, microfinance, and the politics of development.	Rankin KN	220	2002	*Feminist Economics*,
Performance and governance in microfinance institutions.	Mersland R	215	2009	*Journal of Banking & Finance*
Microfinance mission drift?	Mersland R	212	2010	*World Development*
Teaching entrepreneurship: Impact of business training on microfinance clients and institutions.	Karlan D	205	2011	*Review of Economics and Statistics*
Six randomized evaluations of microcredit: Introduction and further steps.	Banerjee	201	2015	*American Economic Journal: Applied*

RETRACTED

### 4.4 Most productive sources

Table 3 listed the top 10 sources of productivity. Only 350 of the 1429 published articles are found in indexed journals. Only 10 journals, however, contain 25 % of all publications published in the same field. This section lists studies that have productive sources linked to microfinance journals.

**Table 3:** Most productive sources.

Sources	Articles
Enterprise Development and Microfinance	68
World Development	59
Journal of International Development	49
Small Enterprise Development	38
Savings and Development	29
Strategic Change	27
Journal of Development Studies	23
Development in Practice	21
Applied Economics	18
International Journal of Social Economics	18

### 4.5 Highly contributive authors

Table 4 lists the ten most well-known authors in microfinance. These authors have written articles that examine microfinance theory from all angles and give a thorough overview of the pertinent literature. The individual contributions of authors may be seen in their papers; hence it is important to highlight their research endeavors. Mersland R. published the most articles (38) on microfinance research during the period 1996 to 2020, followed by Hudon M. (21) and Hartarska V. (16). Based on their contributions, the remaining authors are likewise listed in the table in descending order.

**Table 4:** Highly contributive authors.

Authors	Articles	Authors	Articles
Mersland R	38	Johnson S	11
Hudon M	21	Mia Ma	11
Hartarska V	16	Copestake J	9
Beisland La	13	Hermes N	9
Ashta A	11	Kar Ak	9

### 4.6 Most productive COUNTRIES

The most productive nations in terms of publication are listed in this section. The top 10 most productive countries in the field of microfinance are listed in Table 5 together with the total and average article citation values. It lists the nations in order of highest to lowest total number of citations and papers published. According to citation analysis, the USA receives the most citations, followed by the UK and Norway. Out of 10271 citations, 4700 were from the USA, making it the top research country. Table 5 shows that some nations obtained fewer citations overall but high article citation value which are Japan (260-14), Canada (634-28), and Norway (861-33) respectively. In contrast to other nations that produced more publications but obtained fewer citations, it shows that these nations published fewer articles but received substantial citations. Norway only produced 26 publications, yet those 26 articles garnered an impressive 861 citations. India published 84 articles but only garnered a relatively small number of citations compared to Norway, Belgium, Canada, and Australia. Additionally, it shows that these nations published high-quality microfinance papers rather than quantity. In comparison to other countries, the table indicates that the above countries were able to discover the true potential of the Microfinance and contributed research.

RETRACTED

**Table 5:** Author affiliated COUNTRIES.

Country	Articles	Country	Total Citations	Average Article Citations
USA	183	USA	4700	25.683
India	84	United Kingdom	1433	18.139
United Kingdom	79	Norway	861	33.115
Malaysia	38	Belgium	819	26.419
Belgium	31	Canada	634	28.818
France	31	Australia	475	17.593
Australia	27	India	435	5.179
Norway	26	France	358	11.548
Germany	24	Spain	296	12.87
Spain	23	Japan	260	14.444

The nation's interest in microfinance research is depicted in Fig. 2. Blue is the color used to represent international cooperation between nations. The darker blue indicates more frequent international cooperation. The chart shows that the United States, followed by the United Kingdom, has been the most cooperative country in publishing research on microfinance. Belgium, Norway, the Netherlands, and Australia are among the countries that actively cooperate with other nations. It shows that India and Malaysia are the two most cooperative nations in Asia. It suggests that international collaborations will be able to boost the number of high-quality publications relative to those produced by a single nation.

**Fig. 2:** Countries collaboration chart..

### 4.7 Corresponsding author’s country

Table 6 and Fig. 3display the authors' national affiliations, which aid in understanding the contributions made by various nations and the international cooperation of researchers. The USA is the nation with the most articles written. The SCP (Single Country Publication) shows that the USA followed by India are single leading publication countries. The list of ten SCP countries is displayed in the table in descending order. The MCP (Multiple Country publication) ratios of USA is 18.5 %, meaning 81.5. % of published publications have authors from other nations, as opposed to 18.5 % of articles with USA authors alone. The other top five nations are Canada, Australia, Korea, Taiwan, and Australia. It suggests that these nations have made a major contribution to Microfinance research.

RETRACTED

**Table 6:** Corresponding author’s country.

Country	Articles	SCP	MCP	MCP Ratio
USA	183	149	34	0.1858
India	84	79	5	0.0595
United Kingdom	79	56	23	0.2911
Malaysia	38	28	10	0.2632
Belgium	31	17	14	0.4516
France	31	18	13	0.4194
Australia	27	21	6	0.2222
Norway	26	16	10	0.3846
Germany	24	18	6	0.25
Spain	23	19	4	0.1739

**Fig. 3:** Countries collaboration metrics

### 4.8 Keywords

The information about the author's keywords, keyword plus, and word cloud is provided in this section. The term "keywords plus" refers to terms or phrases that regularly appear in references inside an article. An increasingly common technique for displaying the knowledge structure of scientific domains is to conduct bibliometric analysis based on literature by examining author keywords and keyword plus.

The list of chosen articles by keyword from 1996 to 2019 have been researched and is shown in the table. For this analysis, the time frame before 1996 has not been taken into account. The majority of the literature according to a bibliometric study of author keywords or keyword plus revolves around the following topics: microfinance institutions, poverty, outreach, microcredit, sustainability, and financial performance. The most popular study locations are in the microfinance hubs of Bangladesh and India. The association between author keywords and keyword plus is also shown in Table 7.

**Table 7:** Most frequently used keywords.

Author Keywords	No	Keywords-Plus (ID)	No
Microfinance	683	Microfinance	587
Microfinance Institutions	122	Credit Provision	114
Poverty	77	Lending Behavior	106
Outreach	61	Financial Services	89
Microcredit	60	Poverty Alleviation	78
Bangladesh	56	India	75
Sustainability	49	Banking	67
India	47	Bangladesh	66
Financial Performance	44	Institutional Framework	60
Efficiency	36	Financial System	57

A word cloud of the keywords used in Microfinance is shown in Fig. 4. The most prominent key words are credit provision, lending behavior, financial services, poverty alleviation, financial system, women status, developing world, financial system, institutional framework, financial provision, sustainability, and empowerment. However, along these general terms other popular keywords include sustainability, financial markets, economic competition, and financial management. India, and Bangladesh are underlined here as being most favored research destination in microfinance. The word cloud shows that microfinance has attracted the attention of researchers in the above fields.

RETRACTED

**Fig. 4:** Word cloud.

Fig. 5 displays the trending topics along with their frequency data for each year between 1999 and 2017. Trending keywords from 1999 to 2003 like "economic factors," "macroeconomic factors," "grameen bank," "financial provision," and "socioeconomic impact" shows that impact studies were carried out all over the world in this period to determine the effects of microfinance on economic and socioeconomic factors. The high frequency in the table suggests that in Asia, India and Bangladesh have been the most popular study destinations for microfinance since 2010. The most popular search terms since 2011 have been credit provision, lending behavior, financial services, poverty alleviation, banking, financial system, institutional framework, women's status, and empowerment.

**Fig. 5:** Trending topics..

### 4.9 Three-Field PLOT

The three-field plot reveals an interesting connection between the three core areas of research. Fig. 6 and Table 8 highlight the associations between top authors, key phrases, and top journals related to microfinance research. The important researchers in the field are shown, together with their most popular search terms and the top journals that publish their work. Researchers may be able to find influential authors about microfinance who can be approached for collaboration using the information offered by the three-field plot. The primary research subfields that can be investigated further can also be determined. Moreover, authors can choose more appropriate journals for publishing based on the data regarding the acceptability evaluated using the three-field plot.

**Fig. 6:** Three-Field plot.

**Table 8:** Collaboration of main authors, main keywords, and main journals.

Main Authors	Main Keywords	Main Journals
Mersland R. (38 Papers)	Microfinance (683 Papers)	Enterprise Development and Microfinance (68 Papers)
Hudon M. (21 Papers)	Microfinance Institutions (122 Papers)	World Development (59 Papers)
Hartarska V. (16 Papers)	Poverty (77 Papers)	Journal of International Development (49 Papers)
Beisland L.A. (13 Papers)	Outreach (61 Papers)	Small Enterprise Development (38 Papers)
Ashta A. (11 Papers)	Microcredit (60 Papers)	Savings and Development (29 Papers)
Johnson S. (11 Papers)	Bangladesh (56 Papers)	Strategic Change (27 Papers)
Mia M.A. (11 Papers)	Sustainability (48 Papers)	Journal of Development Studies (23 Papers)
Copestake J. (9 Papers)	India (47 Papers)	Development in Practice (21 Papers)
Hermes N. (9 Papers)	Financial Performance (43 Papers)	Applied Economics (18 Papers)
Kar A.K. (9 Papers)	Efficiency (36 Papers)	International Journal of Social Economics (18 Papers)
Lensink R. (9 Papers)	Gender (30 Papers)	Humanomics (13 Papers)
Morduch J. (9 Papers)	Performance (30 Papers)	Agricultural Finance Review (12 Papers)
Mori N. (9 Papers)	Islamic Microfinance (29 Papers)	Economic and Political Weekly (12 Papers)
Murshid N.S. (9 Papers)	Entrepreneurship (27 Papers)	Journal of Business Ethics (12 Papers)
Szafarz A. (9 Papers)	Financial Inclusion (27 Papers)	Journal of Development Economics (12 Papers)
Quayes S. (8 Papers)	Poverty Alleviation (27 Papers)	Oxford Development Studies (12 Papers)
Schreiner M. (8 Papers)	Regulation (26 Papers)	Quarterly Review of Economics and Finance (12 Papers)
Serrano-Cinca C. (8 Papers)	Mission Drift (24 Papers)	European Journal of Development Research (11 Papers)
D'espallier B. (7 Papers)	Social Capital (24 Papers)	Ids Bulletin (11 Papers)
Gutiérrez-Nieto B. (7 Papers)	Social Performance (23 Papers)	Asian Social Science (10 Papers)
Marr A. (7 Papers)	Empowerment (22 Papers)	International Journal of Rural Management (10 Papers)
Mosley P. (7 Papers)	Microfinance Institution (22 Papers)	Journal of Developmental Entrepreneurship (10 Papers)
Wijesiri M. (7 Papers)	Women (21 Papers)	Annals of Public and Cooperative Economics (9 Papers)
Wydick B. (7 Papers)	Corporate Governance (20 Papers)	Developing Economies (9 Papers)
Awaworyi Churchill S. (6 Papers)	Poverty Reduction (20 Papers)	Mediterranean Journal of Social Sciences (9 Papers)
Chikalipah S. (6 Papers)	Asia (19 Papers)	Nonprofit and Voluntary Sector Quarterly (9 Papers)
Dorfleitner G. (6 Papers)	Ghana (19 Papers)	Perspectives on Global Development and Technology (9 Papers)
Musshoff O. (6 Papers)	Governance (19 Papers)	Development Policy Review (8 Papers)
Nadolnyak D. (6 Papers)	Data Envelopment Analysis (17 Papers)	Economic Modelling (8 Papers)
Panda D.K. (6 Papers)	Developing Countries (17 Papers)	Journal of Banking and Finance (8 Papers)

RETRACTED

### 4.10 keyword analysis

Fig. 7 shows the keyword analysis based on term co-occurrence map based on text data. These keywords are either derived from the title and abstract of each publication or taken directly from the article's keyword list [55]. The study used the VOS viewer software and the fraction counting approach based on number of keywords to create this network. The results showed two distinct clusters related to microfinance. The blue cluster shows that the keyword “microfinance” is linked to poverty, social capital, income, woman empowerment, and development, India and Bangladesh. The green cluster represents that the “Microfinance Institution” keyword is associated with sustainability, cost, efficiency, financial performance, and design methodology approach and microfinance sector. The results divide the microfinance research in two clusters of Microfinance impact studies and Microfinance Institutions studies with related keywords.

Fig. 7: Keyword occurrence networks in 1429 articles selected from a survey sample period 1996–2019.

**Fig. 7:** Term CO-OCCURRENCE map based on text data (title & abstract).

## 5 Summary and direction for further research

The study examined 1429 publications by applying bibliometric analysis and network analysis methods and techniques, Publications from the past 25 years from 1996 to 2019 that have been indexed in the Scopus database are considered. In a nutshell, it represents what has been done and what could be done in future by researchers and academicians. The word cloud and keyword analysis show Microfinance research focused on only developing world particularly Asian countries like India, Bangladesh, Malaysia, and a few African countries. The great success of these projects in developing countries has motivated wealthier countries to imitate them. Additionally, policy makers' interest in microfinance programs has prompted academics to conduct additional research. Therefore, an increase in academic research must be accompanied by a review of the academic literature. This assessment is an important part of the research process, as it enables the identification and classification of the literature, as well as identifying trends and open avenues for scholarly creation. Therefore, the study highlights the summary of literature in Microfinance by representing trends and patterns of Microfinance research related to topmost cited articles, highly productive sources, countries, authors, journals as well as collaboration network of authors and countries. Credit Provision, Lending Behavior, Financial Services, Poverty Alleviation, Indian Banking, Financial System, Institutional Framework, Women Status, and Empowerment have been the most popular Microfinance topics since 2011. Most of the literature on microfinance revolves around the following topics: microfinance institutions, poverty, outreach, microcredit, sustainability, and financial performance, according to result of author keywords or keyword plus. The most popular study locations are Bangladesh and India. The main keyword and keyword analysis based on term co-occurrence map shows that the microfinance research is divided into two clusters. First cluster is of Microfinance impact studies on i.e. (Poverty 77 papers, Micro credit 60 papers, Gender 30 papers, Islamic Microfinance 29 papers, Entrepreneurship 27 papers, financial inclusion 27 papers, social capital 24 papers and Empowerment 22 papers, corporate governance 20 papers). The second cluster is of Microfinance Institutions (MFIs) studies with related keywords i.e. outreach 61 papers, Sustainability 48 papers, financial performance 43 papers, efficiency 36 papers, Mission drift 24 papers, Data Envelopment analysis 17 papers. A detailed overview of the most important studies is summarized in the findings, which would be helpful to academicians interested in microfinance research.

RETRACTED

Based on the result of bibliometric analysis it could be recommended that in future researchers can focus on the developed world. The impact studies of microfinance show mixed result of microfinance on social and economic performance factors. Comparative research are recommended on loan lending models and governance. Research investigating funding landscape, product development, pricing models and strategies at Micro Finance Institutions has been remaining a challenge for academics in the fields of marketing and fintech. Exploring the role of Islamic Microfinance in supporting sustainability and addressing social and environmental issues can provide important insights. Many MFIs are very successful and compete with incumbent financial institutions. In the future, therefore, scholars can focus on comparing MFI performance with that of other financial institutions. In addition, future research may focus on MFIs efficiency and financial sustainability with large sample size including latest data and all relevant databases. However, the study's analysis tools were limited to bibliometric and network analysis. The study is restricted to 1429 microfinance articles from the Scopus database, which were published from 1996 to 2019 in the past 25 years. This may have led to the skipping of other relevant literature and important issues in microfinance in other databases. Moreover, extending the sample size up to 2022 and other relevant databases will cover more dynamics and give more valuable information to researchers. To address these unresolved challenges, we need to develop pertinent strategies, identify relevant tools and techniques, and explore all databases.

## Funding statement

This work is not supported by any organization/university.

## Data availability statement

Data included in article/supplementary material/referenced in article.

## Additional information

No additional information is available for this paper.

## CRediT authorship contribution statement

**Kashif Beg:** Writing – review & editing, Writing – original draft, Visualization, Validation, Supervision, Software, Resources, Project administration, Methodology, Formal analysis, Data curation, Conceptualization. **B. padmapriya:** Writing – review & editing, Visualization, Validation, Supervision, Software, Resources, Project administration, Methodology, Investigation, Formal analysis, Conceptualization. **Syed Noorul Shajar:** Conceptualization, Data curation, Formal analysis, Funding acquisition, Investigation, Methodology, Project administration, Resources, Software, Supervision, Validation, Visualization, Writing – original draft, Writing – review & editing. **Md. Moneef Ahmad:** Writing – review & editing, Visualization, Validation, Supervision, Software, Methodology, Investigation, Formal analysis, Conceptualization. **Abdul Ghani Faiyyaz:** Writing – review & editing, Visualization, Supervision, Software, Resources, Project administration, Methodology, Investigation, Formal analysis, Data curation, Conceptualization.

RETRACTED

## Declaration of competing interest

The authors declare the following financial interests/personal relationships which may be considered as potential competing interests:Kashif Beg reports administrative support was provided by 10.13039/501100004728VIT University AP. Dr Kashif Beg reports a relationship with VIT University AP that includes: employment. If there are other authors, they declare that they have no known competing financial interests or personal relationships that could have appeared to influence the work reported in this paper.
